RETRACTED

# Effects of Anesthetics on Proliferation and Apoptosis of Drug-Resistant Human Colon Cancer Cells

**DOI:** 10.1155/2022/4080585

**Published:** 2022-08-04

**Authors:** Chunrong Tang, Shengdan Fu, Dongsheng She, Juan Zhou, Weixia Su, Tao Zeng

**Affiliations:** ^1^Department of Anesthesiology, Hubei Songzi People's Hospital, Songzi, 434200 Hubei, China; ^2^Obstetrics and Gynecology Department, Hubei Songzi People's Hospital, Songzi, 434200 Hubei, China; ^3^Anorectal, Hubei Songzi People's Hospital, Songzi, 434200 Hubei, China; ^4^Obstetrics Department, Hubei Songzi People's Hospital, Songzi, 434200 Hubei, China

## Abstract

In recent years, people's living standards are getting higher and higher, and life pressure is also increasing, and there are also many problems in eating habits. This is also the direct cause of colon cancer. The aim of this paper was to investigate whether anesthetic drugs could positively affect the proliferation and apoptosis of colon cancer cells. In this paper, the significance of anesthetic drugs is proposed, and an artificial neural network algorithm based on artificial intelligence is proposed. It is well known that artificial neural networks play an important role in medicine. The experimental results of this paper show that the incidence of colon cancer in 2020 will be in the range of 5%-35%, and the incidence of colon cancer in 2021 will be in the range of 7%-30%. While colon cancer rates in 2021 do not appear to be as high as colon cancer rates in 2020, they are generally much higher than colon cancer rates in 2020. It can be seen that as the population ages, the number of colon cancer patients is increasing due to the lack of emphasis on health. This also means that the incidence of colon cancer is getting higher and higher, and traditional drug chemotherapy has been unable to play a good role in inhibiting the proliferation of colon cancer cells. Therefore, this paper investigated the effects of anesthetic drugs on the proliferation and apoptosis of human colon cancer cells.

## 1. Introduction

There are many functions of anesthesia, which can not only make the patient not have pain during the operation but also make the patient not have anxiety and tension during the operation. Now in surgery, it is impossible to imagine what it would be like without anesthesia. If there is no anesthesia drug, what kind of painful ordeal it is for the patient who is going to have the operation: the heart-piercing howl and the bone-piercing feeling. The effect of the doctor's operation will also be greatly reduced, and countless patients die tragically on the operating table. These tragedies were quite normal before the invention of narcotics. The discovery of anesthetics has relieved human suffering, saved more patients' lives, improved human survival ability and quality of life, and benefited future generations by benefiting the human body itself.

RETRACTED

The incidence of colon cancer varies according to region, age, lifestyle, and gender. The regions with high incidence of colon cancer are in developed countries such as Western Europe and North America, and the regions with low incidence are in Africa and Asia. The incidence of colon cancer is higher in men than in women, which may be related to ethnicity, living habits, patterns of work and rest, and type of diet. In addition, studies have shown that the incidence of colorectal cancer increases year by year with age, which may be related to the increase in the incidence of colorectal cancer in China.

The innovations of this paper are as follows: (1) this paper introduces the theoretical knowledge of propofol and nanocapsule preparations and colon cancer. And the artificial intelligence-based neural network algorithm was used to analyze the importance of neural network algorithm in the study of nanocapsule preparations on the proliferation and apoptosis of human colon cancer cells. (2) This paper expounds the artificial intelligence-based neural network algorithm. Through experiments, it was found that the artificial intelligence-based neural network algorithm can effectively analyze the effects of nanocapsules containing propofol anesthetics on the proliferation and apoptosis of human colon cancer cells.

## 2. Related Work

With the improvement of people's living standards in recent years, the importance of physical health is also increasing. Hsiao et al. found that circular RNAs (circRNAs) are a class of noncoding RNAs whose functions are mostly unknown. Some studies suggest that circRNAs may be involved in the pathogenesis of diseases, but there is little direct evidence. Here, he describes the functional role of a novel encoding in colon cancer (CRC), some of which have been quantitatively validated. The experimental results suggest that the novel code exerts its function by regulating a subset of oncogenes. Although he proposed a new type of coding and also drew experimental conclusions, the whole experimental process was not reflected, so the authenticity of his conclusions could not be confirmed [1]. Lee et al. found that although the clinical treatment of colon cancer often does not take into account the primary tumor site, left- and right-sided colon cancers have distinct clinical and biological characteristics. Gene expression analysis further revealed distinct biological subtypes of colon cancer (CRC), identifying 4 shared molecular subtypes. Importantly, these subtypes were distributed differently between right and left CRCs. He has been emphasizing that the characteristics of left- and right-sided colon cancer are different, but there is no specific explanation for the difference [2]. Fukui found that medical researchers prepared bioderived nanocapsules, known as liposome capsules, based on the concept of polyelectrolytes. This approach allows the selection of a wide variety of polymers, from synthetic polymers to biologically derived polymers such as polypeptides and polysaccharides. The resulting nanocapsules exhibited excellent properties, including mechanical strength, controlled release of substances, and enhanced cell membrane permeability. Although he proposed the advantages of nanocapsules, there is no experiment to prove whether its advantages are reliable [3]. Gong et al. discovered an image change detection method based on deep learning, which completes the detection of changed and unchanged regions by designing a deep neural network. Mainly, the trained deep neural network is used to generate the change detection map directly from the two images, which can avoid the influence of the difference image on the change detection result. Learning algorithms for deep architectures include unsupervised learning and supervised learning [4]. Alanis presents the results of the use of recurrent neural networks and their application in electricity price forecasting and an artificial neural network trained by an algorithm based on the extended Kalman filter. Finally, he demonstrates the applicability of the proposed forecasting scheme by using European power system data and forward forecasting. Although he proposed that neural network algorithms can be applied to electricity forecasting, he did not mention how neural networks could be applied to electricity [5]. Perna and Rocca proposed a strategy for choosing the hidden layer size in a feedforward neural network model. What they present is a comparison of a given loss function based on the out-of-sample predictive power of different models. To overcome the problem of data breaches, they extended and modified the scheme based on the use of reality checks. It allows to choose the parsimonious neural network model with the highest prediction accuracy. Although they explained different models, they did not demonstrate the model experimentally [6]. Zhang et al. studied the delay-dependent stability of neural networks, and they considered more information about the activation function and delay upper bound of delayed neural networks. At the same time, they review and compare the most common techniques for dealing with derivatives by introducing relaxation matrices. It was finally found that the introduced relaxation matrix played an important role in reducing conservatism, but they did not give a specific description of the comparisons he made [7]. Chen et al. found that long noncoding RNA is involved in the tumorigenesis of various cancers; however, its role in colon cancer tumorigenesis has not been fully elucidated. Their research shows a potential relationship between RNA and vitamin D receptor signaling. Considering the critical role of signaling in the physiology and pathology of colonic epithelial cells, the correlation between RNA and signaling may have an important role in the development of colon cancer. But they did not explain what role the correlation between RNA and signaling plays [8].

RETRACTED

## 3. Artificial Neural Network Method

### 3.1. Basic Concepts of Colon Cancer

Propofol, a short-acting intravenous anesthetic, is used for the induction and maintenance of general anesthesia. It is often used at the same time as epidural or spinal anesthesia, as well as with analgesics, muscle relaxants, and inhalation anesthetics. Colorectal cancer (CRC), also known as colorectal cancer, is a malignant lesion that occurs in colorectal epithelial cells under the action of various adverse pathogenic factors such as genetics or the environment. This may be due to the continuous improvement of China's economic level; people's living standards have been greatly improved, followed by great changes in people's life and diet [9], thereby laying a health hazard to the occurrence and development of colon cancer. Signs of colon cancer are shown in Figure 1.

As shown in Figure 1, according to statistics, in 2008, there were 1.2 million new colon cancer patients every year in the world, and its mortality accounted for 8% of all malignant tumors. In recent years, colon cancer has developed into one of the most common digestive tract malignant tumors [10].

There are many reasons for the occurrence and development of colon cancer. Studies have shown that the occurrence of colon cancer is caused by the combined influence of heredity and the environment. Among them, the environmental factor is the dominant factor, about 80%. Environmental factors include many aspects, such as lifestyle, mental and psychological factors, dietary structure, and eating habits [11]. Among them, the effects of dietary intervention on colon cancer are more studied. Some studies have suggested that long-term intake of dietary fiber can change the network structure of intestinal flora in vivo. This will affect the gene expression of colon cancer in the process of occurrence and development, which will affect the occurrence of colon cancer to a certain extent [12].

RETRACTED

### 3.2. Narcotic Drugs Containing Propofol Anesthetics

#### 3.2.1. Nanocapsule Preparation

Nanodrug carriers are usually made from natural or synthetic polymeric materials. According to various preparation techniques and materials, it can be divided into nanoparticles, lipid nanoparticles, nanoemulsions, nanocolloids, etc. The advantages of nanodrug carriers are as follows: control the invasion of drugs into specific target organs or target cells and target drug delivery; prolonged drug action time and slow drug release; improved formulation stability and oral biodiversity; and biodegradable, nontoxic, or less toxic carrier materials [13]. The schematic diagram of the nanodrug carrier is shown in Figure 2.

As shown in Figure 2, with the rapid development of nanotechnology, nanomaterials have attracted much attention in the research of tumor diagnosis and treatment. Because of their good biocompatibility, they are often used as nanodrug delivery carrier materials. Compared with normal cells, biotin is essential for tumor proliferation and biotin receptors are highly overexpressed on the surface of tumor cells. It can be used as a ligand in combination with nanodrugs to actively target tumors [14].

#### 3.2.2. Propofol

In order to find a drug with fast anesthesia effect, short maintenance time, no accumulation after repeated administration, and no excitatory effect during induction, anesthesia, and recovery, physicians found that propofol was ideal during screening. Since propofol was listed in the UK in 1986, it has been widely used abroad in recent years and has been widely used in clinical practice [15]. It includes induction and maintenance of anesthesia; even in larger abdominal surgery, the effect is also very good; spinal anesthesia can also be used.

Propofol has the following advantages: rapid onset and complete effect; stable anesthesia, induction and maintenance; rapid recovery after long-term large-scale medication; during the recovery period, the recovery of mental activity is fast, and the incidence of nausea after wood is low; the pharmacokinetic parameters are stable; and it is easy to adjust the drug delivery rate, in order to achieve the purpose of different medicinal techniques: no accumulation in the body and no organ toxicity [16]. The disadvantages are as follows: high-dose use can inhibit breathing; the blood pressure lowering effect and the heart rate increasing effect of the drug are greater than those of thiopental sodium; and the injection site is slightly painful.

The core of chemotherapy is to enter the blood circulation through oral absorption or injection and then be transported to the lesion through the blood circulation to exert its effect. During this process, the distribution of many chemotherapeutic drugs in the body cannot be controlled. As a result, the chemotherapeutic drugs that reach the diseased tissue are effective, and the chemotherapeutic drugs that reach the normal tissue cause toxic side effects.

RETRACTED

In order to overcome many shortcomings of previous chemotherapy, pharmacists have conducted many studies from a new perspective, hoping to improve existing cancer chemotherapy drugs [17].

#### 3.2.3. The Effect of Narcotic Drugs Encapsulating Propofol Anesthetics

“Composite drug carrier” is a concept of “top-down” drug carrier construction proposed in recent years, which is characterized by selecting natural biomaterials with various properties according to various therapeutic needs in order to be compatible with existing nanoformulations. The narcotic drugs is shown in Figure 3.

As shown in Figure 3, the application of nanotechnology in the field of pharmaceuticals is based on the fact that it can change the microscopic state of the drug, thereby changing the biopharmaceutical properties of the drug, with excellent properties of reducing drug toxicity and side effects [18].

1. Promote apoptosis and inhibit the proliferation of colon cancer cells

A major feature of colon cancer cells is their ability to escape programmed cell death or apoptosis. Apoptosis of body cells is a complex dynamic process, regulated by both proapoptotic genes and antiapoptotic genes. The immortal proliferation of colon cancer cells caused by a variety of gene mutations can disturb this balance [19]. The combined use of apoptosis-inducing genes in colon cancer cells and proapoptotic drugs is expected to be a novel colon cancer therapy. Induction of apoptosis depends on the expression of tumor suppressor genes.

(2) Reverse drug resistance genes

Long-term chemotherapy may make patients resistant to chemotherapy drugs, and drug resistance is a major obstacle to the treatment of colon cancer. Therefore, if the related proteins of colon cancer drug resistance gene are reversed, drug resistance can be largely reversed, and combined with chemotherapy drugs, the effect of chemotherapy can be improved [20].

### 3.3. Feature Gene Selection of Cancer Cells Based on Artificial Neural Network

The neuron of an artificial neural network is a simple processing unit. Processing units can be arbitrary objects, such as functions, characters, concepts, and some meaningful abstract patterns. Neurons are divided into three types: input neurons, hidden neurons, and output neurons, which can imitate the information storage and processing functions in the human brain nervous system at different levels and degrees [21]. The application areas of neural networks are shown in Figure 4.

RETRACTED

As shown in Figure 4, so it has characteristics such as parallelism, structural variability, and nonlinearity; artificial neural network is an academic topic that includes artificial intelligence, computer science, neuroscience, thinking science, and other fields. It has been evaluated by many scholars, applied to many research fields, and achieved many epoch-making results.

### 3.4. Feature Extraction Based on Flexible Neural Tree

Neural tree is proposed to solve the problem of automatic design of artificial neural network. It is an intelligent computing system similar to artificial neural network, which uses evolutionary computing to assist its structure and parameter optimization. The flexible neural tree model is composed of two types of instruction sets: functional instruction set (denoted by *F*) and terminal instruction set (denoted by *T*). The functional instruction set is composed of nonleaf nodes in the flexible neural tree, and the terminal nodes are composed of input features. The flexible neural tree model can be expressed as

(1) $$\begin{array}{c} S=F\cup T=\left\{+2,+3,\cdots ,+N\right\}\cup \left\{a_{1},a_{2},\cdots ,+a_{n}\right\}, \end{array}$$

where +*i*(*i* = 2, 3, ⋯, *N*) represents a nonleaf node with *i* parameters (or branches), and *a*_1_, *a*_2_, ⋯, *a*_*n*_ represents a leaf node without any parameters. The flexible neuron operator and flexible neural tree are shown in Figure 5.

As shown in Figure 5, this is a flexible neuron operator and flexible neural tree. In the process of creating a flexible neural tree structure, the Gaussian distribution function is often used as the excitation function for nonleaf nodes. If +*i*(*i* = 2, 3, ⋯, *N*) is selected, the weight *w*_*i*_ and the two parameters *a*_*i*_ and *b*_*i*_ in the excitation function are randomly generated at the same time. The excitation function of nonleaf nodes is as follows:

(2) $$\begin{array}{c} f\left(a,a_{i},b_{i}\right)=e^{-\left(1/2\right){\left(\left(a-a_{i}\right)/b_{i}\right)}^{2}} \end{array}$$

In a neural network, there is a functional relationship between the input and output of the hidden layer and output layer nodes, and this function is called the excitation function. The formula for calculating the total excitation result of neuron + *i* is as follows:

(3) $$\begin{array}{c} {\text{net}}_{i}=\overset{i}{\underset{j=1}{\sum }}w_{j}\times a_{j}, \end{array}$$

where *a*_*j*_(*i* = 2, 3, ⋯, *j*) represents each input of node + *I*.

The optimization of flexible neural tree mainly includes optimization of tree structure and optimization of parameters. The optimization of the tree structure is actually a process of feature selection.

RETRACTED

Supposing *c*_*ij*_ represents the classification result of the classifier composed of category *i*(*i* = 1, 2, ⋯, *k*) and category *j*(*j* = 1, 2, ⋯, *k*) and *i* ≠ *j*, if *c*_*ij*_=1, it means that the test sample is divided into category *i*, otherwise it is 0.

Majority voting is the most widely used in the field of ensemble classification. The main idea is as follows: first, each subclassifier classifies and judges the test samples, then votes, and finally calculates the votes of each category, and the category with the most votes is the predicted category of the test sample. The number of votes is calculated as

(4) $$\begin{array}{c} V\left(i\right)=\underset{1\leq j}{\sum }c_{ij}. \end{array}$$

Then, the judgment of which category the test sample *z* finally belongs to is as follows:

(5) $$\begin{array}{c} c=\arg\max V\left(i\right). \end{array}$$

The advantage of this method is that it does not require the participation of additional computation and knowledge, and the disadvantage is relatively obvious. The majority voting method assigns the same weight to each subclassifier, which will increase the impact of poor-performing individuals on the overall performance of the ensemble.

The Bayesian combination method is different from the voting method that uses the combination of the classification results of each subclassifier *c*_*ij*_ to decide the ensemble result. The Bayesian combinatorial approach evaluates each subclassifier and derives the probability that the final classification result may be erroneous. The specific calculation description is shown in the following formula:

(6) $$\begin{array}{c} c=\arg\max\left\{\overset{k}{\underset{j=1}{\prod }}P\left(z\left|c_{ij}\right.\right)\right\}. \end{array}$$

It can be seen from formula (6) that the Bayesian combination method requires the participation of prior knowledge.

### 3.5. BP Neural Network Method

Neurons are neuron cells, which are the most basic structural and functional units of the nervous system, divided into two parts: cell body and protrusion. The cell body is composed of the nucleus, cell membrane, and cytoplasm and has the function of connecting and integrating input information and outgoing information. There are two types of protrusions: dendrites and axons. Artificial neural network is widely used in various medical fields, and its popularization and application are inseparable from the development of neural network. The neurons of biological nervous system are connected by synapses. The connection method is shown in Figure 6.

RETRACTED

As shown in Figure 6, by defining *a* = [*a*_1_, *a*_2_, ⋯, *a*_*n*_] to represent the axonal output and *w* = [*w*_*i*1_, *w*_*i*2_, ⋯, *w*_in_] to represent the connection strength, the output of a neuron can be expressed as

(7) $$\begin{array}{c} b=f\left(\overset{R}{\underset{i=1}{\sum }}w_{i}a_{i}-\theta \right). \end{array}$$

BP neural network is a feedforward network, usually composed of an input layer, a hidden layer, and an output layer, and its development is based on the development of biological neural network. It can simulate the stimulation of the brain, respond to external stimuli, and adapt to changes in the experimental environment through continuous learning and error correction. It has strong adaptive ability, self-learning ability, and generalization function. Samples are trained and output, analyze the internal relationship between input and output, find the law, and use this law to process and model complex data. The BP neural network is shown in Figure 7.

As shown in Figure 7, the logsig function is the sigmoid function in logistic regression. The BP neuron is similar to other neurons, but the difference is that the transfer function of the BP neuron is a nonlinear function, the most commonly used functions are the logsig function and the tansig function, and the output layer adopts a linear function. Its output is as follows:

(8) $$\begin{array}{c} a=\log\text{sig}\left(wp+b\right) \end{array}$$

The logarithmic sigmoid transfer function logsig is as follows:

(9) $$\begin{array}{c} \text{logsig}\left(n\right)=\frac{1}{1+e^{-n}} \end{array}$$

The hyperbolic tangent sigmoid function tansig is as follows:

(10) $$\begin{array}{c} \tan\text{sig}\left(n\right)=\frac{e^{n}-e^{-n}}{e^{n}+e^{-n}} \end{array}$$

The disadvantages are as follows: there is the phenomenon of majority coercion, that is, the external cost; compared with the unanimous agreement rule, the choice behavior of a single participant is no longer decisive, which affects the enthusiasm of individuals to participate in voting and ultimately affects the real preference display; there is a “voting paradox.” Due to various factors such as the complexity of the problem, the slowness of the convergence rate, the network being restricted to a minimum value, and the vibration of the learning process, the choice of algorithm is often a matter of concern. The logsig and tansig functions are shown in Figure 8.

As shown in Figure 8, in the training of neural network, the problem of “overfitting” may occur. That is, the sample error within the training group is small, but the new sample data error outside the training group is very large. Therefore, in order to improve the generalization ability of the network, it is usually necessary to adjust the size of the network to make it “appropriate.”

RETRACTED

The basic idea of the normalization method is to modify the network error performance function, which is as follows:

(11) $$\begin{array}{c} F=\text{mse}=\frac{1}{N}\overset{N}{\underset{i=1}{\sum }}{\left(e_{i}\right)}^{2}=\frac{1}{N}\overset{N}{\underset{i=1}{\sum }}{\left(t_{i}-a_{i}\right)}^{2} \end{array}$$

If a parameter is added, which includes the mean square value of the network weights and thresholds and the error performance function is corrected by this parameter, the generalization ability of the network can be improved, which is as follows:

(12) $$\begin{array}{c} \text{Msereg}=\gamma \cdot \text{mse}+\left(1-\gamma \right)\text{msw} \end{array}$$

*γ* in the formula is the error performance adjustment rate.

The BP network for pattern recognition classification can be designed with reference to the following formula:

(13) $$\begin{array}{c} n=\sqrt{n_{i}+n_{0}}+a \end{array}$$

Among them, *n*_*i*_ is the number of input nodes, and *n*_0_ is the number of output nodes. The transfer function in the BP network usually adopts the *S*- (sigmoid-) type function, which is as follows:

(14) $$\begin{array}{c} f\left(a\right)=\frac{1}{1+e^{-a}} \end{array}$$

There is another independent variable *a*_1_, *a*_2_..*a*_*m*_, denoted *P* = *P*(*B* = 1/*a*_1_, *a*_2_, ⋯*a*_*m*_), and the logistic regression model can be expressed as

(15) $$\begin{array}{c} P=\frac{1}{1+\exp\left[-\left(\beta_{0}+\beta_{1}a_{1}+\beta_{2}a_{2}+\cdots +\beta_{m}a_{m}\right)\right]} \end{array}$$

*β*_0_ is a constant term, and *β*_1_, *β*_2_, ⋯, *β*_*m*_ is a regression coefficient.

Cox proportional hazards model is an analysis method generally used in survival analysis and is a multivariate survival analysis method. Its expressions are formula (16) and formula (17):

(16) $$\begin{array}{c} H\left(t\left|A\right.\right)=h\left(t\right)\exp\left(A\beta \right), \end{array}$$

(17) $$\begin{array}{c} \text{HR}=\frac{h\left(t\left|a_{1}\right.\right)}{h\left(t\left|a_{2}\right.\right)}=\frac{h_{0}\left(t\right)\exp\left(A_{1}\beta \right)}{h_{0}\left(t\right)\exp\left(A_{2}\beta \right)} \end{array}$$

For different individuals *A*_1_ and *A*_2_, the hazard ratio is independent of the baseline hazard function and does not change with time *t*.

In recent years, the research of artificial neural network has attracted more and more attention, and it has been widely used in clinical medicine in recent years due to the superior self-organization adaptability, learning ability, and excellent analysis characteristics of complex nonlinear systems. Disease diagnosis, survival prediction, disease screening, and many other aspects are used.

RETRACTED

## 4. Experiments and Analysis of Colon Cancer Development

### 4.1. Development and Pathogenesis of Colon Cancer

With the birth of human beings, various diseases have emerged, and human beings have begun to suffer from the harm and invasion of these diseases. Among them, cancer poses the greatest threat to human health. In medicine, when a patient is diagnosed with cancer, it is usually in the middle and late stages of cancer, which also leads to a very high mortality rate for cancer patients. Among cancer patients, middle-aged people have the highest mortality rate. There are currently more than 10 million cancer patients worldwide. The incidence of colon cancer from 2020 to 2021 is shown in Figure 9.

As shown in Figure 9, with the change of dietary structure, the incidence of common intestinal diseases such as colitis and colon cancer is increasing year by year. Due to the repeated and long course of these diseases and the fact that it is difficult to detect, it has laid a great hidden danger to people's health.

At present, the number of colon cancer patients is still on the rise. Therefore, colon cancer has become a major killer that threatens human life, and the treatment and prevention of colon cancer have also become the focus of scientists in the fields of medicine and biology around the world. So far, the pathological mechanism and treatment options of colon cancer are still poorly understood. The characteristics of colon cancer are shown in Figure 10.

As shown in Figure 10, at the same time, research into drugs to prevent or treat colon cancer has been considerably limited. The diversity of colon cancer is about 60%, and the complexity is about 75%. The key to this series of problems is that cancer is a very complex and intractable disease in medicine. It not only has many types and complex structures, but also, cancer cells are easy to spread and metastasize.

In recent years, with the development of China's economic level, changes in living habits, changes in diet and lifestyle, and the acceleration of population aging, the incidence and mortality of colorectal cancer in China have gradually increased. It is one of the major malignant tumors that endanger people's life and health. Risk factors for colon cancer are shown in Figure 11.

As shown in Figure 11, the risk factors for colon cancer include gender, age, environmental factors, obesity, diabetes, lack of exercise, smoking, and alcohol dependence. Therefore, colon cancer is one of the important diseases that threaten public health in China. Colon cancer is a malignant tumor of the colon. Once it occurs, it will seriously affect the health of the patient. If not treated in time, the disease of colon cancer will further aggravate and even threaten the life of the patient.

RETRACTED

### 4.2. Experimental Analysis of Narcotic Drugs Containing Propofol Anesthetics

Among the current treatment methods for colon cancer, the most important method is chemotherapy, which has huge toxic and side effects, and many chemotherapy drugs, especially natural products, have low water solubility and must be administered by injection. To overcome the many defects of chemotherapeutic drugs, nanoformulations came into being. The many properties of nanoformulations have greatly improved the clinical application status of some anticancer drugs, and many types of nanoformulations have been successfully marketed.

With the deepening of research, the advantages of nanoformulations in the treatment of colon cancer have been widely recognized. However, due to the inherent properties of this drug, injections are often the only available route of administration, and oral administration of injections is important to improve treatment compliance and reduce treatment costs. The significance of the narcotic drugs encapsulating propofol anesthetics is shown in Table 1.

As shown in Table 1, when the contained nanometer is 5 nm, the rate of cancer cell proliferation is 10%, and when the contained nanometer is 20 nm, the rate of cancer cell proliferation is 2%. This study observed the effect of different concentrations of narcotic drugs encapsulating propofol anesthetics on the proliferation of human colorectal cancer cells. The results showed that the nanocapsule preparation encapsulated with propofol anesthetic drug can promote the apoptosis of human colon cancer cells and has a significant inhibitory effect on cell proliferation, and the inhibitory effect is stronger with the increase of drug concentration.

### 4.3. Experiments on Flexible Neural Tree and Feature Extraction Method

In order to compare with the previous research results, the LOOCV cross-validation method is used to process the data set in the experiment. The so-called LOOCV verification method is each time a sample is taken from the overall sample as a test sample and all other samples are used as training samples. There are 10 experiments carried out for each sample set, and then, the average of the 10 classification results was calculated as the final experimental result. In this paper, the experimental analysis of flexible neural tree and feature extraction method and the hybrid feature extraction method combining the two is simplified, as shown in Tables 2 and 3.

As shown in Tables 2 and 3 , the classification accuracy of the test set is 79.04%, and the classification accuracy of the training set is 79.04%, indicating that the method in this paper is effective. It is the eigengenes extracted by the feature extraction method that affect the classification accuracy in this experiment—the hybrid feature extraction method, which proves that the eigengenes extracted by the flexible and flexible neural tree can improve the classification accuracy. The flexible and flexible neural tree can perform both feature extraction and classification. All the above data show that the method proposed in this paper is more effective than other methods.

RETRACTED

## 5. Conclusions

With the development of society, various diseases also emerge in an endless stream. Among them, colon cancer is a kind of cancer that is more troublesome to people's physical and mental health, and the incidence rate is also rising. Therefore, it is very necessary to inhibit colon cancer cell proliferation and promote colon cancer cell apoptosis. This paper mainly studies the effects of anesthetics on the proliferation and apoptosis of colon cancer cells. It is found that anesthetics can inhibit the proliferation of colon cancer cells and promote cell apoptosis. This paper adopts artificial neural network algorithm. In recent years, scholars have begun to explore the application of neural networks in medical research and have achieved many promising results. However, injectable drug delivery remains an insurmountable chasm. Research on narcotic drugs is in the ascendant. How to make the emerging anesthetics with many advantages further practical is a topic of great research value. Therefore, this paper has certain significance for the study of anesthetics.

## Figures and Tables

**Figure 1:** Signs of colon cancer.

**Figure 2:** Schematic diagram of nanodrug carrier.

**Figure 3:** Narcotic drugs.

**Figure 4:** Application areas of neural networks.

**Figure 5:** Flexible neuron operator and flexible neural tree.

**Figure 6:** Schematic diagram of biological neurons.

**Figure 7:** BP neural network.

**Figure 8:** Logsig and tansig functions.

**Figure 9:** Incidence of colon cancer, 2020-2021.

**Figure 10:** Features of colon cancer.

**Figure 11:** Risk factors for colon cancer.

**Table 1:** Inhibition rate and promotion rate of propofol-encapsulated narcotic drugs on human colorectal cancer cells.

Concentration	Cell proliferation	Apoptosis
5 nm	10%	37%
10 nm	5%	48%
15 nm	3%	55%
20 nm	2%	59%

**Table 2:** Experimental results of the three methods in the first 5 experiments.

Method	Test set classification accuracy (%)	Running time (seconds)
Flexible neural tree	57.73	242.8
Feature extraction	56.90	689.4
Hybrid feature extraction	79.04	135.7

RETRACTED

**Table 3:** Experimental results of the three methods in the last 5 experiments.

Method	Test set classification accuracy (%)	Running time (seconds)
Flexible neural tree	50.64	280.4
Feature extraction	53.05	785.0
Hybrid feature extraction	80.52	153.2

## Data Availability

The data that support the findings of this study are available from the corresponding author upon reasonable request.
